The article "A Pilot Study of Compensatory Strategies for Reach-to-Grasp-Pen in Patients with Stroke" was published in 2022. Journal: Appl Bionics Biomech.

# A Pilot Study of Compensatory Strategies for Reach-to-Grasp-Pen in Patients with Stroke

**DOI:** 10.1155/2022/6933043

**Published:** 2022-11-11

**Authors:** Qiurong Xie, Bo Sheng, Jia Huang, Qi Zhang, Yanxin Zhang

**Affiliations:** ^1^College of Rehabilitation Medicine, Fujian University of Traditional Chinese Medicine, Fuzhou 350122, Fujian, China; ^2^Key Laboratory of Orthopedics & Traumatology of Traditional Chinese Medicine and Rehabilitation (Fujian University of TCM), Ministry of Education, Fuzhou, China; ^3^School of Mechatronic Engineering and Automation, Shanghai University, Shanghai 200444, China; ^4^Department of Exercise Sciences, The University of Auckland, Newmarket, Auckland 1142, New Zealand

## Abstract

Coordinated reaching and grasping movements may be impaired in patients with poststroke hemiplegia. Patients frequently adopt compensatory strategies, which require investigation. This pilot study used kinematic parameters to examine compensatory strategies by assessing the reach-to-grasp-pen movements in patients with stroke and unaffected participants. Twelve patients with stroke with mild impairment (45.16 ± 12.62 years, 2.41 ± 1.97 months), twelve with moderate impairment (50.41 ± 12.92 years, 3.83 ± 3.58 months), and ten healthy individuals (20.6 ± 0.69 years) performed a reach-to-grasp-pen task. Kinematics parameters of upper limb and fingers, such as movement time, number of movement units, index of curvature, spectral arc length, trunk forward transition, trunk lateral transition, elbow extension, shoulder flexion, shoulder abduction, trunk rotation, arm-plane angle, the joint angles of interphalangeal joints of the thumb, index, middle, ring, and little fingers were examined in the study. These parameters were evaluated with two Microsoft Azure Kinect and Leap Motion, which belong to markerless motion capture systems. Patients with stroke showed longer reaching movement time, less smooth movement trajectories, and more trunk rotation (*P* < 0.05). In patients with stroke, the metacarpophalangeal joint (MCP) and proximal interphalangeal joint (PIP) of the thumb were flexed in the starting position; the MCP and PIP joints of the index finger in the stroke group were more extended during pen grasp; the range of motion of the MCP of the middle finger and the PIP joints of the middle, ring, and little fingers became greater, suggesting a larger peak aperture (*P* < 0.05). The more significant extension was observed in the index finger at the end of the grasp, suggesting inadequate flexion (*P* < 0.05). In clinical practice, the reach-to-grasp-pen task using markless sensing technology can effectively distinguish patients with stroke from healthy individuals and evaluate the recovery and compensation strategies of upper limb and hand functions. It can potentially become an evaluation tool in hospital and community scenes. Accurate identification of abnormal trunk, arm, and finger strategies is crucial for therapists to develop targeted upper limb treatment methods and evaluate treatment effects.

## 1. Introduction

Upper extremity dysfunction in patients with stroke may lead to dependence on daily life activities (ADL) and a poor quality of life. The ability to perform ADLs is highly dependent on hand function [1], and patients often have impairments in grip strength, power, and overall function of the hand that make it difficult to perform daily tasks, severely impairing their ability to perform functional activities independently and reducing their quality of life [2]. Studies have shown that patients with hemiplegia have slower, less fluid movements, lower accuracy, and more significant motor variability in reaching tasks compared to healthy individuals [3]. Compensatory movements are usually observed in patients with stroke; for example, some use excessive trunk and shoulder displacement during reaching, called compensations, to adapt movements in a task-dependent manner [4].

The movement of patients with stroke is characterized by flexor synergy. The abnormal synergy patterns of shoulder and elbow joints reduce the available degrees of freedom, leading to poor spatiotemporal inter-joint coordination of reaching movements [5] and, consequently, more torsional and less smooth endpoint movements. The grasping function is also affected in patients with stroke. During grasping tasks, patients with stroke tend to have slower hand movements, a prolonged terminal phase of reaching and grasping earlier, larger grip apertures, and increased path length of the hand [6]. They may also show impaired grip strength during grasping and lifting [7]. Patients with stroke have been shown to use various compensatory strategies to improve grasping function, such as reduced finger abduction, proximal interphalangeal joint (PIP) flexion, and metacarpophalangeal joint (MCP) extension during object grasping.

Unfortunately, hand function recovery is among the most challenging tasks in stroke rehabilitation. Restoring upper limb and hand functions requires therapeutic intervention to reduce movement disorders. Due to the lack of precise hand function evaluation methods and targeted intervention, the intervention effect is poor. At present, standard clinical evaluation relies on clinical scales. Although they can reflect motor quality, their accuracy and precision are insufficient. At the first consensus meeting of the stroke recovery and rehabilitation roundtable (SRRR) group, experts suggested that quantitative movement analysis of functional tasks may help determine the motor pattern and whether the improvement of the upper limb and hand function is due to appropriate motor recovery or compensation pattern [8]. The markerless sensing technology accurately and effectively measures motion and distinguishes neural changes related to motion recovery and compensation strategies, reflecting the quality of motion more accurately and comprehensively. Markerless motion capture equipment was used in the study to track anatomical landmark positions using computer vision technology, and no physical markers would be needed. Moreover, the most common movement in kinematic studies is pointing or reaching. Previous studies have assessed upper limb or hand function separately, and very few studies have considered both upper limb and hand function in a single functional task [9]. Thus, from a clinical perspective, studying functional task(s) involving both upper limb and hand function may offer more excellent and valuable information about the whole upper limb motor control.

This pilot study aimed to identify and quantify upper extremity and hand function compensatory strategies through a reach-to-grasp-pen task in patients with stroke and to explore the use of that reach-to-grasp-pen task as movement for use in routine upper extremity rehabilitation assessment. It hypothesized that common compensatory strategies (flexor synergy, excessive trunk motion, and finger coordination) can be identified during a reach-to-grasp-pen task and that these strategies are affected by the level of disease.

## 2. Materials and Methods

### 2.1. Participant

Twenty-four patients with stroke and ten healthy individuals were recruited between August 1, 2020 and December 1, 2020. All participants' characteristics are shown in Table 1. Patients with hemiplegia and healthy individuals were recruited to participate in the study. The following study criteria rendered patients with stroke eligible for inclusion: first single cerebrovascular accident; hemorrhagic or ischemic; any time after stroke; left or right hemisphere affected; age between 18 and 90 years; able to sit for at least 5 min without trunk support; able to perform a sitting reach-to-grasp-pen task with the affected hand; Modified Ashworth Scale (MAS) score of hand flexor ≤3; and no history of complex medical conditions such as cardiac, pulmonary, or orthopedic disease. Moderate upper extremity impairment was defined as an FMA-UE motor score (Fugl–Meyer Assessment of Upper Extremity motor function) between 32 and 57 and mild impairment between 58 and 65 [10]. Patients were excluded if their medical history indicated: severe cognitive impairment (minimum mental status examination score <24 [11]), severe aphasia with comprehension impairment or severe neglect.

The study was conducted in the occupational therapy department of Fujian Provincial Rehabilitation Hospital, and an occupational therapist referred patients. The healthy group was recruited at Fujian University of Traditional Chinese Medicine. The Ethics Review Committee approved the study protocol of Fujian Provincial Rehabilitation Hospital (No. 2021KY-005-02), and all subjects provided informed consent according to the Declaration of Helsinki.

### 2.2. Experimental Procedure

Patients underwent standard neurological and musculoskeletal assessments before the experiment. These included the FMA-UE motor score [12] and the modified Ashworth scale [13] and modified Barthel index (MBI) [14]. During the experiment, participants sat in a straight-backed chair, with a seat 45 cm from the ground, in front of a table 75 cm from the ground, with their backs supported but unrestrained. In the initial position, the participant placed their test hand on the table with the forearm pronation, fingers in a fist, and the wrist line near the table's edge. The upper arm was in a neutral position with the elbow flexed at ∼90°. The participant's other hand rested on their knee. Visual inspection was performed to ensure that each trial participant had the same starting hand position. The penholder and pen, about 5 cm^2^ wide and 5 cm high, were placed on the table in front of the subject. The distance was determined according to the length of the subject's active extended arm (i.e., from the medial axilla to the distal wrist crease). In the study, the healthy individuals used the dominant hands to complete the task.

The reach-to-grasp-pen task comprised reaching, grasping the pen from the penholder, putting down the pen slowly and steadily, and returning the hand to its initial position (see Figure 1). Participants were asked to sit against the back of the chair throughout the task but were not restricted in their sitting position and could perform compensatory movements if needed (see Figure 2). They were asked to begin the task following verbal instruction from the tester, at which point they started the task at a comfortable self-paced speed. Each participant completed the task five times, and each task was recorded.

Two Microsoft Azure Kinect cameras (Microsoft, Redmond, WA, USA) and one Leap Motion (LMC, San Francisco, CA, USA) were markerless motion capture systems for 3D motion analysis of the torso and upper extremities and hands during the reach-to-grasp-pen task. Before data collection, Microsoft Azure Kinect cameras were placed on a tripod 1 m above the ground. The distance between the two Kinect cameras was 3 m, as shown in Figure 2. Microsoft Azure Kinect cameras record 3D coordinate data of 25 anatomical landmarks at a sampling frequency of 30 Hz, including head, neck, shoulder, spine, left and right shoulders, left and right elbows, left and right wrists, left and right hands, left and right fingertips, left and right thumbs, middle ridge, left and right hips, left and right knees, left and right ankles, and left and right feet. Leap motion was used to collect hand position information of hand activities and was placed on the table 0.5 m from the subjects. Leap motion can calculate and record each finger joint's flexion/extension angle and horizontal abduction angles between two adjacent fingers (except the thumb) (see Figure 3). The 3D coordinate positions of the markers were calculated immediately, throughout the motion, with high spatial resolution camera units (1 MP Time-of-flight Depth camera, 12 MP CMOS sensor rolling shutter RGB camera). The system was calibrated before each measurement, and data were automatically collected by the Kinect SDK (Microsoft Azure Kinect SDK 1.2, Microsoft). The captured data were transferred to MATLAB software (MathWorks Inc., Natick, MA, USA) for custom analysis.

### 2.3. Data Analysis

This study recorded the three-dimensional coordinates of anatomical markers recognized from the Kinect system bone model during the task. Local segment coordinates, including the torso and upper arm, are established, and each segment coordinate is based on global coordinates. For Kinect upper limb evaluation system, the measured node space position is used as input, and the joint angle and space-time parameters are calculated by the developed unmarked point motion analysis system. A Butterworth low-pass filter with a cutoff frequency of 6 Hz is used. Microsoft Azure Kinect can measure *XYZ* coordinate data of 25 joints of the body. The study used kinematic data from ten joints, including the spine, shoulder/middle, left/right shoulder, left/elbow, left/wrist, and left/right hand. Each repetition segments the original data and is then filtered by singular spectrum analysis to reduce the impact of noise. Apply the data analysis software to calculate the kinematic index according to the filtered data (see Figures 4 and 5). Then, our customized upper limb kinematics calculates the three Euler angles of shoulder rotation for the Microsoft Azure Kinect system, which follow the sequence of flexion (+)/extension (−), adduction (+)/abduction (−), and internal rotation (+)/external rotation (−). Elbow flexion is calculated using trigonometric functions from the position data of shoulderright, elbowright, and wristright. The formula for the three Euler angular velocities is as follows (*ZXY* rotation sequence):

(1) $$\begin{array}{c} \omega_{f}=-\sin\;\theta_{3}\theta_{2}+\cos\;\theta_{3}\cos\;\theta_{2}\theta_{1}, \end{array}$$

(2) $$\begin{array}{c} \omega_{a}=\cos\;\theta_{3}\theta_{2}+\sin\;\theta_{3}\cos\;\theta_{2}\theta_{1}, \end{array}$$

(3) $$\begin{array}{c} \omega_{i}=\theta_{3}-\sin\;\theta_{2}\theta_{1}, \end{array}$$

where *θ*_1_, *θ*_2_, and *θ*_3_ represent the rotation angle around the *Z*, *X*, and *Y*, respectively. *ω*_*f*_, *ω*_*a*_, and *ω*_*i*_ represent the angular velocities of shoulder flexion, adduction, and pronation, respectively.

The specific movements assessed in the reach movements mainly include shoulder flexion, elbow extension, and wrist extension. The specific movements assessed in the grasping movement include wrist extension, finger extension, and finger flexion. The endpoint parameters were calculated based on the hand markers. Each kinematic variable was calculated as the average of all motion segments for the entire task. Movement time was the time required to complete a movement segment; the number of movement units (NMU) were calculated according to the number of velocity peaks in a motion segment and used to measure movement smoothness. A motion unit included acceleration, velocity peaks, and deceleration. The velocity distribution graph established the local minimum and maximum values to define a motion unit. When the difference between the minimum and the next maximum value exceeded a critical value of 20 mm/s, it was considered a velocity peak. In addition, the time between two subsequent peaks had to be at least 150 ms. These peaks reflected the repeated acceleration and deceleration on arrival, reflecting the smoothness and efficiency of the motion. The curvature index was calculated as the ratio between the total terminal path length and the straight line connecting the initial and final positions. This parameter reflected the efficiency of the motion.

Elbow and shoulder joint angles were calculated by the dot product of the vectors, defined by the coordinates of the adjacent marker points. Shoulder flexion was defined as the angle between the vector of the elbow joint and the ipsilateral shoulder marker and the vertical vector from the shoulder marker to the hip (i.e., between the straight lines through the torso). The horizontal shoulder abduction/adduction angle was measured by the angle between the vector formed by the elbow joint and the ipsilateral shoulder marker and the angle between the two shoulder crest markers. The elbow joint angle was defined by the vector formed between the wrist joint and the elbow marker and between the elbow joint and the ipsilateral scapular marker.

In order to determine the possible compensatory movements of adjacent segments, trunk displacement and shoulder peak displacement were calculated. Torso axial rotation was defined as the rotation angle of the point sagittal line in the horizontal plane projection vector of both shoulders. Trunk flexion was defined as the maximum forward displacement from the initial position at the sternal point in the sagittal plane.

After collecting Leap Motion data and using the developed data processing software to determine the finger bone vector, the included angle between finger joints can be calculated through the following formula *θ*_1_, *θ*_2_, and *θ*_3_ (see Figure 3).

(4) $$\begin{array}{c} \theta_{1}=\text{arccos}\left(\frac{\overset{⟶}{WM}\cdot \overset{⟶}{MP}}{\overset{⟶}{\left|WM\right|}\cdot \overset{⟶}{\left|MP\right|}}\right), \end{array}$$

(5) $$\begin{array}{c} \theta_{2}=\text{arccos}\left(\frac{\overset{⟶}{MP}\cdot \overset{⟶}{PD}}{\overset{⟶}{\left|MP\right|}\cdot \overset{⟶}{\left|PD\right|}}\right), \end{array}$$

(6) $$\begin{array}{c} \theta_{3}=\text{arccos}\left(\frac{\overset{⟶}{PD}\cdot \overset{⟶}{DT}}{\overset{⟶}{\left|PD\right|}\cdot \overset{⟶}{\left|DT\right|}}\right). \end{array}$$

The excursion of each finger, i.e., the extent to which the thumb, index finger, middle finger, ring finger, and little finger could be flexed and extended—including the MCP, PIP, and distal interphalangeal (DIP) joints—was measured in the reaching and grasping task. The range of motion of fingers was calculated as difference between the minimum and maximum values in finger angle data (see Figure 3).

### 2.4. Statistical Analysis

Statistical analysis was performed using IBM SPSS 20.0 (IBM Corp, Armonk, NY, USA). In the analysis of kinematic data, the mean of five records was used in the statistical calculations. The measures were expressed as mean ± standard deviation, and the counts were expressed as rates or percentage composition ratios. One-way analysis of variance was used to determine whether there were any significant differences between the means of the three groups, with the least significant difference (LSD) test between groups when differences were significant and general linear model correction analysis when baseline levels were not equal. When the data were not normally distributed and homoscedastic, the Kruskal–Wallis test (a nonparametric test) was used to examine the significant differences among these three groups. All statistical tests were performed using two-sided tests, and *P* values ≤0.05 were considered statistically significant for the differences tested.

## 3. Results

Demographic data and clinical characteristics of 24 patients with stroke and 10 healthy individuals are displayed in Table 1.

Twelve patients with stroke with mild impairment (45.16 ±12.62 years, 2.41 ± 1.97 months) and twelve with moderate impairment (50.41 ± 12.92 years, 3.83 ± 3.58 months) completed all clinical and kinematic assessments. Ten healthy individuals (20.6 ± 0.69 years) completed kinematic assessments. Participants with stroke had mild levels of upper limb (UL) motor impairment (FMA = 60.33 ± 2.70), modified Ashworth scale (0.25 ± 0.45), and MBI (81.25 ± 15.53). Participants with stroke had moderate levels of UL motor impairment (FMA = 44.08 ± 10.62), modified Ashworth scale (0.91 ± 0.66), and MBI (78.75 ± 16.65). All subjects were right-hand dominant. The hand dominance was not significantly different between participants with stroke and healthy groups, but persons with stroke were older than healthy controls.

### 3.1. Comparison of Kinematic Characteristics of the Reaching and Grasping Pencil Task

Statistically significant differences in curvature index (*F*=4.645, *P*=0.017), spectral arc length (*F*=12.471, *P* ≤ 0.001), lateral trunk displacement (*F*=4.303, *P*=0.022), elbow extension (*F*=6.242, *P*=0.005), shoulder flexion (*F*=3.879, *P* ≤ 0.001), shoulder abduction (*F*=4.549, *P* ≤ 0.001), forward trunk displacement (*Z*=21.282, *P* ≤ 0.001), movement time (*Z*=20.583, *P* ≤ 0.001), and movement units (*Z*=17.799, *P* ≤ 0.001) were identified in the these three groups. The stroke group's trunk rotation (*F*=0.183, *P*=0.833) and arm plane angle (*F*=0.247, *P*=0.783) showed no significant differences compared with the healthy group. These are shown in Table 2. Compared with the healthy group, the mild stroke group had longer movement time (*P*=0.001), more motor units (*P*=0.028), greater curvature index (*P*=0.017), and smaller length of the spectral arc (*P* ≤ 0.001), less elbow extension (*P*=0.048), less forward trunk displacement (*P* ≤ 0.001), and more horizontal displacement (*P*=0.006). The moderate stroke group had longer movement time (*P* ≤ 0.001), more motor units (*P* ≤ 0.001), greater curvature index (*P*=0.035), and smaller spectral arc length (*P*=0.017), less elbow extension (*P*=0.001), less shoulder flexion (*P*=0.009), more shoulder abduction (*P*=0.046) and less forward displacement of the trunk (*P*=0.005) than those of the healthy group.

### 3.2. Comparison of Joint Angles of Pen Grasping Strategies

To describe the pen grasping strategies of patients and healthy individuals, the differences in the MCP and interphalangeal (IP) joints of the thumb, and the joint angles of the MCP, PIP, and DIP of the index, middle, ring, and little fingers at the beginning and end of the grasp were all examined.

At the grasp start position, there was a significant difference in the thumb MCP (*F*=4.645, *P*=0.018) and thumb PIP (*F*=4.727, *P*=0.017) among these three groups. The thumb MCP was more flexed (*P*=0.05), and the PIP was more flexed (*P*=0.005) in the mild stroke group.

At the grasp end position, there was a significant difference in the index MCP (*F*=4.455, *P*=0.021), index PIP (*F*=3.441, *P*=0.046), and little MCP (*Z*=6.779, *P*=0.034) among these three groups. Compared with the healthy group, there was less MCP (*P*=0.006) and PIP flexion (*P*=0.017) in the index finger and less MCP flexion (*P*=0.045) in the little finger in the moderate stroke group. The remaining joint angles showed no significant difference (*P* > 0.05). Further details can be found in Table 3.

### 3.3. Change in Joint Angle during Grasping Task

In terms of maximum flexion values, there was no statistical difference between the stroke and healthy groups, as shown in Table 4.

In terms of maximum extension values, there were significant differences in the index finger MCP (*F*=3.562, *P*=0.041) and PIP (*F*=4.112, *P*=0.027) among these three groups. The mild stroke group had smaller maximum extension values for index finger MCP (*P*=0.017) and PIP (*P*=0.017) than the healthy group. In the moderate stroke group, the maximum extension values of the index finger MCP (*P*=0.048) and PIP (*P*=0.019) were smaller than those of the healthy group (see Table 4).

For the range of motion, there were significant differences in the middle MCP (*F*=3.086, *P*=0.034) and PIP (*F*=4.469, *P*=0.020), ring PIP (*F*=6.814, *P*=0.004), and little PIP (*F*=7.587, *P*=0.002) among these three groups. In the mild stroke group, MCP (*P*=0.010) and PIP (*P*=0.006) were greater in the middle finger, PIP (*P*=0.001) in the ring finger, and PIP (*P*=0.001) in the little finger than those of healthy group. The moderate stroke group had more significant PIP (*P*=0.012) in the ring finger and greater PIP (*P*=0.007) in the little finger than in the healthy group. The overall range of motion was greater in the stroke group than in the healthy group, although this difference was not statistically significant (Table 4). Furthermore, the standard deviation was greater in the stroke group, with more significant individual differences. The standard deviation of movement was smaller in the healthy group, and consistency was better in the healthy group.

## 4. Discussion

To the best of the authors' knowledge, this is the first study to extensively examine the reach-to-grasp-pen task in patients with stroke with mild-to-moderate upper extremity motor deficits, aiming to investigate the kinematic characteristics of the upper extremity, trunk, and hand during the task. The results indicate that the reach-to-grasp-pen task can reveal compensatory strategies and differentiate between patients with stroke. The reach-to-grasp-pen task can thus be considered an appropriate tool for assessing the upper extremity in individuals with stroke.

### 4.1. Reaching and Grasping Task Performance

In the present study, the stroke group showed minor elbow extension and shoulder flexion than healthy individuals. Compensatory movements were observed, including excessive shoulder abduction and trunk forward movement. Previous studies have also shown that patients with chronic moderate to severe stroke may have up to 33% increased trunk motion and a combination of shoulder abduction and elevation (i.e., arm plane) motion, even when reaching a target near the arm or the arm [15]. Santos et al. [16] analyzed the movement strategies of patients with stroke to accomplish the task of drinking, and the affected upper extremity showed more scapular protraction and ipsilateral trunk lateral flexion than healthy subjects throughout the drinking process; this was particularly pronounced during the two phases at the beginning of the movement and when the hand reached the cup. Merdler et al. [17] found higher arm abduction and minor elbow extension in all target directions in the stroke group compared with the healthy group; the arm plane angle tended to be higher in the moderate to severe stroke group.

For the grasping behavior, the thumb flexion appeared hypertonic in the stroke group at the onset. The thumb MCP and PIP were more flexed in the stroke group (*P* < 0.05), suggesting the presence of thumb flexion muscle tone in the stroke group. Clinically, patients with stroke with moderate-to-severe hand injury usually present with bending of the thumb to the palm and bending of the fingers to the thumb. Hyperexcitability of the musculi flexor pollicis longus (FPL), which manifests as spasticity, excessive synergistic activity, and delayed relaxation, is thought to be responsible for this phenomenon [18]. In the present study, the flexion tone of the thumb did not seem to affect the patients' pen grasp performance since no significant differences in MCP joint activity were observed during the task undertaken.

The stroke group did not seem able to control the scaling of the peak finger aperture during the reach-and-grasp-pen task; the maximum extension values of the MCP and PIP of the index finger were smaller in the stroke group than in the healthy group (*P* < 0.05), and each joint of the index finger was less flexed and more extended in the stroke group. In addition, the range of motion of the MCP and PIP joints of the middle, ring, and little fingers was greater in the stroke group (*P* < 0.05). This may be due to the lack of motor control in the stroke group, resulting in a larger range of motion. These findings suggest that the fingers of the stroke group could not control the size of the aperture, and therefore, the peak aperture was larger. A grasping motion requires precise planning and execution of hand movement toward the object and prediction of the grasping aperture for object properties. Reaching and grasping movements performed after a stroke are characterized by slow hand transmission, slow grasping apertures, inaccurate scaling of peak grasping apertures, and decoupling of spatiotemporal coordination between hand transmission and grasping aperture components [6].

The ability to open the fingers during the grasping aperture component of the grasping action is altered after stroke due to the impairment of coordination and timely activation of finger muscles in patients with stroke and with the activation of more proximal muscles in the transport component of the hand, making it difficult to open the fingers accurately when approaching the grasped object. In particular, the problem of activating the finger extensors and coordinating the muscle activity between the finger flexors and extensors leads to a highly variable grasp aperture [6]. In the present study, the larger aperture may have resulted from a limited ability to flex the index finger or from a deterioration in motor control of the fingers.

In the grasp end position, the index finger MCP and PIP were less flexed in the stroke group (*P* < 0.05); that is, in a more extended position, suggesting a problem with index finger opposition, flexion function, or just a problem with the gripping strategy. One study showed that patients with stroke used more MCPs for grasping [19]. This differs from the present study, possibly because Raghavan and colleagues used the task of grasping a rectangular wooden block, while the present study used a pen grasp task. Another study has proposed that mild and moderate impairments influenced patients' grasp preferences. Those with moderate motor impairment primarily used the affected upper extremity and full hand grasp, whereas those with mild impairment tended to use a finger grasp [20]. However, in our study, no features of full-handed grasping were found. It is, however, possible that the patients included in this study were relatively mildly impaired. In addition, there were significant differences between stroke groups and healthy groups. The other two groups differed significantly from the healthy group, so this task can distinguish healthy people from patients with stroke. Future studies can recruit more patients and age-sex-matched healthy people to observe whether this task can distinguish patients with different severity.

Clinically, patients with low muscle tone cannot complete functional reaching and grasping movements. The goal of treatment in this period is to induce positive movements, and the therapist will not evaluate their fine movements. Therefore, we did not recruit patients with hypotonia in the flaccid paralysis period in this study but recruited patients with spasticity who could complete reaching and grasping movements.

### 4.2. Underlying Neurophysiological Mechanisms of Performance Deficits

In the present study, the stroke group had more shoulder abduction and scapular elevation, possibly due to coactivation of the trapezius muscle or coactivation of the anterior, middle, and posterior deltoid muscles. A previous study found that the motor unit recruitment level of the upper trapezius during reaching was more significant in the hemiplegic side of patients with stroke than in healthy subjects. The anterior deltoid/superior trapezius work ratio was less than in healthy subjects, which suggests that the compensatory contraction of the upper trapezius muscle in the hemiplegic side of patients was enhanced during the forward flexion reaching task [21]. In another study, the same was found for the electromyogram (EMG) signal of the reaching action, where patients required more compensation from the trapezius muscle relative to the healthy group, and the contraction strength of other muscles was generally smaller. The lack of elbow extension in the stroke group may be due to insufficient activation of the triceps muscle. Pan et al. [22] studied the changes in muscle synergy during active reaching movements in subacute stroke survivors. They observed reduced activation of the triceps, coactivation of the trapezius and deltoid muscles, and increased activation of the pectoralis major in the stroke group. Levin et al. [23] found that stroke may lead to a limitation of reciprocal inhibition and excessive coactivation of the agonist–antagonist muscles, resulting in coactivation of the biceps and triceps. This may be due to a defect in tension stretch reflex (spatial) threshold regulation in both muscle groups, leading to limited elbow extension.

Results from the current study show that the motor control of the fingers of patients with stroke during pen grasp was reduced, and the peak aperture was larger than was the case for the healthy group. Poor motor control may be related to the loss of independent finger control [24]. Impaired independence of all fingers, including the thumb, in patients with moderate hand motor impairment due to subcortical stroke is an essential cause of deficits in hand motor control [24–27]. The lack of independence is attributed to many factors, including peripheral connective tissue connections between the fingers, multifidus extrinsic hand muscles, and overlapping cortical representation of the fingers [28]. Overall, how the fingers are innervated is primarily determined by central neural factors [29]. With infarction in the middle cerebral artery, the loss of higher motor planning and sensorimotor integration greatly disrupts fine force production, especially during finger independence [30]. Secondary degeneration of the corticospinal tract and loss of motor units in spinal cord segments occur in the days and weeks following ischemic injury, leading to permanent deficits in motor performance that can result in poor finger coordination and impaired hand function [31].

Sensory deficits may also lead to reduced finger control. Umeki et al. [32] conducted sensory training to enhance finger discrimination in patients and found that the mean change in tactile pressure threshold was significantly greater in the experimental group than in the healthy group. The reduction in manipulation time required for handling small balls and small metal discs observed in the experimental group was significantly greater than in the healthy group. The results suggest that a sensory training program that enhances finger discrimination helps to improve not only the sensory function but also the hand function of patients with stroke and that the improvement of somatosensory deficits after stroke reflects the control of finger movements. Sensory deficits after stroke include tactile loss and protective and proprioceptive loss. Sensory feedback information is critical because the amount of sensory feedback information generated by cutaneous sensory receptors affects the control of motor function (requiring precision).

### 4.3. Clinical Implications

Studies have shown that patients with stroke may adopt atypical compensatory movements to perform tasks [33], and this phenomenon was also identified in the current study. Evidence suggests that the continued use of these compensatory modalities may be detrimental to true rehabilitation [34]. Replicating the correct kinematics is vital for training because restoring preinjury kinematic movements, rather than using an altered (compensatory) kinematic approach, is fundamental to true rehabilitation [35]. Therefore, it is crucial to identify compensatory patterns.

Previous studies have identified differences between healthy individuals and patients with stroke in the upper extremity, trunk, and hand kinematics using reach-to-grasp and grasp tasks, respectively. This study extends previous findings on hand function deficits in neurological patients. Our results suggest that patients with stroke present with compensatory reach-and-grasp-pen strategies, abnormal upper extremity and trunk kinematic metrics, and poor hand motor control. The reach-and-grasp-pen task used in the study could be a valuable supplement to the current strategy of measuring hand compensation. It could be used to measure motor quality (i.e., trunk and arm joint displacement and intersegmental coordination) and endpoint performance (i.e., spatiotemporal quality of whole arm movement) [36], which is in line with the recent proposal arising from the first consensus meeting of the SRRR to assess upper extremity motor quality by functional activity [8]. In clinical practice, the reach-to-grasp-pen task can be used to evaluate the recovery and compensation strategies of patients with stroke's upper limb and hand function, which helps evaluate the clinical efficacy of treatment methods and judge the neurological mechanism of functional improvement. In the subsequent research, we will continue to collect extensive sample data to form an intelligent evaluation system for stroke upper limb function to automatically identify defective dysfunction, which is more conducive to the clinical application of occupational therapists.

### 4.4. Study Limitations

The current study has several limitations. First, only mild-to-moderate patients with stroke were recruited, and the study results cannot be generalized to patients with severe stroke. Furthermore, the age and gender were not matched between the groups. Second, EMG data were not recorded. Future work could combine information regarding brain networks, muscle networks, and muscle synergy to understand the neurophysiological mechanisms of the disease better and help therapists improve treatment and rehabilitation programs. Furthermore, we will select age- and gender-matched healthy participants and the population of the specific onset period and age group in the future study.

## 5. Conclusions

The study presented here has found that patients with stroke showed poor endpoint performance and more trunk displacement in the upper extremity during a reach-to-grasp-pen task. There was high thumb flexion tension and poor finger motor control during pen grasp. Impaired upper extremity, hand motor control, and altered reach-to-grasp-pen strategies were found in patients with varying degrees of stroke. The results from our study indicated that the reach-to-grasp-pen task could differentiate patients with stroke from healthy people, which may be considered a standard tool for functional assessment of the upper extremity.

## Figures and Tables

**Figure 1:** Schematic diagram of experimental design.

**Figure 2:** (a) Experimental scenario; (b) a subject (subject08) was performing the reach-to-grasp pen task; (c) Microsoft Azure Kinect data collection software; (d) leap motion data collection software.

**Figure 3:** (a) Microsoft Azure Kinect anatomical landmarks; (b) leap motion finger joints; (c) leap motion finger geometry and the phalangeal joints' declination angle. Metacarpophalangeal, proximal interphalangeal, distal interphalangeal, and fingertip are represented by W, M, P, D, and T, respectively.

**Figure 4:** Microsoft Azure Kinect and leap motion data processing software.

**Figure 5:** Kinematic metrics.

**Table 1:** Characteristics of healthy and stroke subjects.

Characteristic	Healthy group (*n*=10)	Stroke group mild stroke (*n*=12)	Moderate stroke (*n*=12)
Age, years	20.6 ± 0.69	45.16 ± 12.62	50.41 ± 12.92
Gender (female : male), *n*	0 : 10	2 : 10	6 : 6
Side of the lesion (left : right), *n*	N/A	5 : 7	6 : 6
Dominant hand (left : right), *n*	0 : 10	0 : 12	0 : 12
Type of stroke (hemorrhage : infarct), *n*	N/A	5 : 7	6 : 6
Time since stroke, months	N/A	2.41 ± 1.97	3.83 ± 3.58
FMA-UE (/66)			
Total	N/A	60.33 ± 2.70	44.08 ± 10.62
Modified Ashworth scale	N/A	0.25 ± 0.45	0.91 ± 0.66
Modified Barthel index	N/A	81.25 ± 15.53	78.75 ± 16.65

Abbreviations: FMA-UE, upper extremity part of the Fugl–Meyer Motor Assessment (maximal score 66); N/A, not applicable. Mild group: stroke patients with mild motor impairment. Moderate group: stroke patients with moderate motor impairment. Modified Barthel index: Flexor muscle of finger.

**Table 2:** Kinematic characteristics of the reach-to-grasp-pen task in healthy and stroke subjects.

Parameters	Healthy group (*n*=10)	Stroke group mild stroke (*n*=12)	Moderate stroke (*n*=12)	*F*/*Z* value	*P* value
Movement time (s)	1.35 (1.25–1.43)	2.49 (1.89–2.77) ± 0.65^a^	2.65 (2.08–3.37)^a^	20.583	≤0.001
Number of movement unit	1.00 (1.00–1.00)	1.67 (1.50–2.20)^a^	2.50 (2.06–3.80)^a^	17.799	≤0.001
Index of curvature	1.11 ± 0.06	1.20 ± 0.03^a^	1.26 ± 0.33^a^	4.645	0.017
Spectral arc length	−1.51 ± 0.08	−1.60 ± 0.08^a^	−1.71 ± 0.09^a^	12.471	≤0.001
Trunk forward transition (mm)	2.55 (2.26–3.45)	0.20 (0.05–0.49)^a^	0.48 (0.35–0.68)^a^	21.282	≤0.001
Trunk lateral transition (mm)	1.85 ± 1.29	4.06 ± 2.02^a^	3.08 ± 1.80	4.303	0.022
Range of motion (degree)					
Elbow extension	69.23 ± 7.29	58.47 ± 10.22^a^	50.82 ± 16.43^a^	6.242	0.005
Shoulder flexion	54.73 ± 7.12	48.66 ± 9.84	43.11 ± 11.37^a^	3.879	0.031
Shoulder abduction	9.84 ± 3.14	12.85 ± 3.55	17.61 ± 9.22^a^	4.549	0.019
Trunk rotation	14.91 ± 5.21	13.67 ± 4.85	13.49 ± 7.19	0.183	0.833
Arm-plane angle	23.13 ± 6.70	25.43 ± 8.68	23.21 ± 10.61	0.247	0.783

Mild group: stroke patients with mild motor impairment. Moderate group: stroke patients with moderate motor impairment. ^a^Compared with the healthy group, *P* < 0.05. ^b^Compared with the mild group, *P* < 0.05.

**Table 3:** Comparison of finger joint angles at the starting and end positions in grasping tasks in healthy and stroke subjects.

Joint	The initial position of grasping					The end position of grasping				
	Healthy	Mild	Moderate	*F*/*Z* value	*P* value	Healthy	Mild	Moderate	*F*/*Z* value	*P* value
MCP										
Thumb	9.36 ± 4.34	17.18 ± 7.83^a^	13.43 ± 4.65	4.645	0.018	11.51 ± 7.82	9.53 ± 6.71	10.89 ± 4.85	0.254	0.778
Index	50.55 ± 8.68	48.79 ± 13.91	39.06 ± 10.84	3.148	0.058	48.14 ± 7.82	39.03 ± 14.77	31.66 ± 13.79^a^	4.455	0.021
Middle	50.86 ± 6.88	54.90 ± 13.87	43.90 ± 10.26	2.894	0.071	42.93 ± 6.40	45.54 ± 11.92	38.82 ± 20.01	0.451	0.641
Ring	44.78 ± 8.35	49.51 ± 17.57	41.08 ± 14.19	0.994	0.382	53.62 ± 9.28	50.37 ± 15.06	40.23 ± 19.89	2.156	0.134
Little	43.71 ± 7.89	48.79 ± 19.90	41.56 ± 15.26	0.640	0.535	65.34 (60.85–66.85)	63.53 (51.98–70.92)	47.42 (31.95–60.55)^a^	6.779	0.034
PIP										
Thumb	16.67 ± 7.36	28.19 ± 10.60^a^	24.20 ± 7.55	4.727	0.017	19.92 ± 11.69	16.18 ± 10.56	19.52 ± 7.47	0.452	0.641
Index	37.96 ± 10.42	46.30 ± 18.22	37.74 ± 12.61	1.271	0.296	53.40 ± 10.18	42.95 ± 6.89	39.59 ± 17.63^a^	3.441	0.046
Middle	50.06 ± 11.39	58.54 ± 16.39	56.08 ± 13.47	1.009	0.377	54.25 ± 7.39	54.95 ± 10.66	55.39 ± 19.64	0.018	0.982
Ring	50.53 ± 10.39	56.81 ± 18.05	54.16 ± 11.92	0.531	0.593	55.45 ± 5.65	53.52 ± 11.01	50.72 ± 14.44	0.482	0.622
Little	53.65 ± 8.21	57.55 ± 16.06	50.92 ± 10.30	0.832	0.445	48.93 ± 5.44	51.84 ± 9.94	47.14 ± 14.01	0.556	0.579
DIP										
Index	23.66 ± 5.19	30.93 ± 10.67	25.77 ± 7.79	2.169	0.132	39.83 ± 12.56	36.47 ± 14.70	29.92 ± 14.43	1.372	0.269
Middle	34.87 ± 10.61	37.83 ± 7.91	46.72 ± 17.90	2.430	0.106	46.43 ± 6.58	45.88 ± 12.28	44.06 ± 16.47	0.104	0.902
Ring	43.88 ± 12.51	43.59 ± 12.03	49.98 ± 17.08	0.709	0.500	50.28 ± 4.72	51.64 ± 11.11	49.86 ± 18.44	0.057	0.945
Little	48.56 ± 9.97	45.43 ± 14.26	53.78 ± 19.44	0.845	0.440	51.79 ± 8.41	51.89 ± 8.93	53.77 ± 19.13	0.077	0.926

Mild group: stroke patients with mild motor impairment. Moderate group: stroke patients with moderate motor impairment. ^a^Compared with the healthy group, *P* < 0.05. ^b^Compared with the mild group, *P* < 0.05.

**Table 4:** Comparison of maximum flexion values, maximum extension values, and joint range of motion in the stroke and healthy groups.

	Peak flexion, degrees					Peak extension, degrees					Range of motion, degrees				
	Healthy	Mild	Moderate	*F*/*Z* value	*P* value	Healthy	Mild	Moderate	*F*/*Z* value	*P* value	Healthy	Mild	Moderate	*F*/*Z* value	*P* value
MCP															
Thumb	17.16 ± 7.37	21.41 ± 7.31	19.56 ± 6.96	0.913	0.413	3.77 (0.25–6.51)	3.15(0.52–4.72)	4.49 (2.19–7.63)	1.045	0.593	13.64 ± 5.76	17.97 ± 5.87	14.79 ± 5.26	1.687	0.203
Index	56.70 ± 5.25	56.95 ± 9.34	52.31 ± 9.64	1.046	0.364	18.60 ± 6.13	10.80 ± 7.95^a^	12.21 ± 6.94^a^	3.562	0.041	38.09 ± 6.64	46.15 ± 11.72	40.10 ± 9.49	2.034	0.149
Middle	54.62 (51.80– 58.13)	67.77 (65.34–72.45)	54.39 (47.81– 76.78)	4.064	0.131	23.24 ± 9.06	17.91 ± 12.83	18.64 ± 15.36	0.595	0.558	34.28 ± 11.72	48.17 ± 17.70^a^	41.67 ± 11.55	3.806	0.034
Ring	59.29 (56.12–62.90)	68.22 (62.96–72.96)	55.88 (51.06–66.56)	4.506	0.105	25.96 ± 11.96	20.41 ± 15.77	19.85 ± 17.54	0.498	0.613	34.28 ± 11.72	45.40 ± 13.01	39.42 ± 9.29	2.485	0.101
Little	66.24 (64.07–66.89)	69.14 (66.80–72.77)	55.81 (53.09–72.48)	3.486	0.175	26.47 ± 12.30	25.44 ± 18.08	21.31 ± 15.26	0.332	0.720	38.78 ± 11.28	40.44 ± 15.83	40.81 ± 7.41	0.083	0.921
PIP															
Thumb	29.14 ± 10.32	35.11 ± 8.88	32.37 ± 8.03	1.131	0.337	6.45 (0.88–12.71)	3.69 (0.95–7.66)	9.28 (3.72–13.92)	2.057	0.358	22.47 ± 6.81	29.12 ± 7.28	23.21 ± 5.98	3.171	0.057
Index	55.69 ± 8.99	58.01 ± 11.30	53.32 ± 17.24	0.223	0.801	25.40 ± 7.08	18.12 ± 7.76^a^	18.24 ± 4.57^a^	4.112	0.027	30.28 ± 9.03	39.89 ± 10.18	36.07 ± 14.25	1.857	0.174
Middle	62.43 ± 6.91	73.43 ± 9.26	71.11 ± 15.10	2.823	0.076	33.31 ± 9.80	30.68 ± 12.67	33.93 ± 16.30	0.183	0.834	29.12 ± 7.18	42.75 ± 10.36^a^	37.18 ± 12.78	4.469	0.020
Ring	62.52 ± 5.28	70.47 ± 10.56	68.43 ± 8.59	2.180	0.131	38.11 ± 11.09	29.31 ± 14.86	31.49 ± 14.26	1.180	0.322	24.40 ± 8.69	41.16 ± 13.17^a^	36.94 ± 9.66^a^	6.814	0.004
Little	59.27 ± 5.83	67.95 ± 10.44	64.60 ± 2.58	2.712	0.083	36.26 ± 11.14	36.26 ± 11.14	27.45 ± 14.39	1.581	0.223	23.00 ± 6.36	41.01 ± 15.58^a^	37.14 ± 8.72^a^	7.587	0.002
DIP															
Index	41.92 ± 11.87	46.77 ± 12.23	42.07 ± 14.42	0.492	0.616	15.98 ± 4.06	10.95 ± 5.86	11.73 ± 4.14	3.293	0.051	25.94 ± 12.97	35.81 ± 10.23	30.34 ± 14.53	1.597	0.220
Middle	54.48 ± 9.09	63.80 ± 9.32	65.81 ± 15.40	2.750	0.081	23.24 ± 9.06	22.03 ± 11.89	23.99 ± 13.58	0.078	0.925	31.23 ± 14.03	41.77 ± 8.60	41.81 ± 14.44	2.416	0.107
Ring	62.53 ± 7.15	68.20 ± 8.13	70.36 ± 12.28	1.865	0.173	33.03 ± 10.08	26.70 ± 12.24	28.86 ± 14.61	0.686	0.512	29.49 ± 11.19	41.49 ± 11.56	41.49 ± 16.25	2.810	0.077
Little	66.97 ± 4.90	71.81 ± 11.15	73.85 ± 11.50	1.350	0.275	36.78 ± 8.58	31.48 ± 14.87	34.84 ± 14.16	0.452	0.641	30.19 ± 7.83	40.32 ± 12.27	39.00 ± 12.55	2.501	0.099

Mean ± SD of peak flexion, peak extension, and total mean range of motion (flexion minus extension) of the distal interphalangeal (DIP), proximal interphalangeal (PIP) and metacarpophalangeal (MCP) joints of each finger in the healthy group and patients. Mild group: stroke patients with mild motor impairment. Moderate group: stroke patients with moderate motor impairment. ^a^Compared with the healthy group, *P* < 0.05. ^b^Compared with the mild group, *P* < 0.05.

## Data Availability

The datasets used and analyzed during the current study are available from the corresponding author upon reasonable request.
